The article "Significance of Cardiometabolic Index in Predicting Acute Exacerbation of Stable Chronic Obstructive Pulmonary Disease for Clinical Nursing" was retracted in 2023. Reasons: suspected computer-generated content; unreliable results or conclusions; concerns about the data; concerns about the results or conclusions.

# Significance of Cardiometabolic Index in Predicting Acute Exacerbation of Stable Chronic Obstructive Pulmonary Disease for Clinical Nursing

**DOI:** 10.1155/2022/7539520

**Published:** 2022-11-07

**Authors:** Ruqiao Luo, You Xia, Shengtao Li, Yinju Ding

**Affiliations:** Department of Emergency, The First Hospital of Changsha, Changsha 410005, Hunan Province, China

## Abstract

**Objective:**

To evaluate the level of cardiometabolic index (CMI) to predict the risk of acute exacerbation in patients with stable chronic obstructive pulmonary disease (COPD), and to provide a basis for early identification and intervention of high-risk patients in clinical nursing work.

**Methods:**

Patients with stable chronic obstructive pulmonary disease who were admitted to the outpatient department of respiratory medicine in a tertiary hospital or followed up after discharge from January to December 2021 were retrospectively selected. CMI was measured and statistical analysis was performed to determine the optimal threshold for predicting acute exacerbation of chronic obstructive pulmonary disease.

**Results:**

A total of 63 patients with chronic obstructive pulmonary disease were enrolled. The median number of episodes in the previous year was 1.00; 44 patients had ≥1 acute exacerbation. The CMI was positively correlated with the frequency of acute exacerbations and the British Medical Research Council (mMRC) score in the previous year, and negatively correlated with the percentage of forced expiratory volume in 1 second to the predicted value (FEV1% PRED). The cut-off point of CMI for predicting acute exacerbations in stable chronic obstructive pulmonary disease patients was 2.05, with a sensitivity of 0.864% and specificity of 0.842%. It is a risk factor for acute exacerbation in COPD patients.

**Conclusion:**

CMI can be used as a biological index to predict acute exacerbation in stable COPD patients. Clinical nursing needs to evaluate patients' CMI and provide personalized nursing intervention for patients with CMI≥2.05.

## 1. Introduction

Chronic obstructive pulmonary disease (COPD) is a common respiratory disease, which is characterized by progressive airflow obstruction, chronic inflammation of the lungs, and the occurrence of persistent symptoms and acute exacerbations [1]. At present, chronic obstructive pulmonary disease (COPD) is highly prevalent, and its morbidity and mortality are both at a high level, and patients are prone to recurrent acute exacerbations of COPD (AECOPD), resulting in worsening of respiratory and systemic symptoms and increased mortality [2]. Statistics show that the number of deaths of COPD patients in China can reach 1 million each year. Therefore, early diagnosis, timely treatment, and accurate assessment of adverse prognostic risk are crucial to improving treatment effect and prognosis [3]. Therefore, it is important to look for indicators that can objectively assess COPD and predict the risk of acute exacerbation and death. In this way, high-risk patients can be identified in advance in nursing work and provide a basis for early clinical intervention.

The article "Significance of Cardiometabolic Index in Predicting Acute Exacerbation of Stable Chronic Obstructive Pulmonary Disease for Clinical Nursing" was retracted in 2023. Reasons: suspected computer-generated content; unreliable results or conclusions; concerns about the data; concerns about the results or conclusions.

Current studies have confirmed that systemic inflammation and oxidative stress are related to COPD disease progression and prognosis [4]. The cardiometabolic index is an indicator of major heart disease. Recent studies suggest that the level of cardiometabolic index in COPD patients is significantly higher than that in healthy controls, while Wakabayashi et al. found that cardiometabolic index is correlated with heart failure in elderly COPD patients [5, 6]. Based on this background, patients with stable COPD who were admitted to the outpatient department of respiratory medicine in a tertiary hospital or followed up after discharge from January to December 2021 were selected as the research objects. To explore the optimal threshold of CMI level for predicting acute exacerbation in stable COPD patients by detecting CMI.

## 2. Methods

### 2.1. Patients and Method

The trial was designed to be an intervention-free retrospective study, with patient data collected between January 2021 and December 2021. In this study, patients admitted to the inpatient department of respiratory medicine and outpatient department of respiratory medicine in The First Hospital of Changsha were screened according to the following inclusion and exclusion criteria. The study was approved by the hospital's Ethics Committee and informed consent was signed by all patients.

#### 2.1.1. Inclusion Criteria

(1) The diagnosis of COPD was based on the Global Initiative for Chronic Obstructive Pulmonary Disease (GOLD) guidelines; (2) age ≥40; (3) no history of respiratory tract infection in recent 4 weeks; (4) did not receive antibiotic treatment or systemic use of glucocorticoids in the last 4 weeks; and (5) informed consent.

#### 2.1.2. Exclusion Criteria

(1) Fever, worsening cough, increased sputum or change of sputum nature, and dyspnea worse than before within 1 month before the test; (2) used intravenous or oral hormones within 1 month prior to participating in the trial; (3) patients with serious cardiovascular and cerebrovascular diseases and other acute or chronic inflammatory diseases; (4) women who are in pregnancy or lactation; and (5) those with mental and behavioral disorders who cannot cooperate to complete the test.

### 2.2. Research Method

The demographic data, smoking status, acute exacerbation frequency of COPD within one year, lung function, and other data of patients were collected from the hospital electronic medical record system. When the subjects were registered, the modified British Medical Research Council (MMRC) Dyspnea Questionnaire was measured, and the cardiac metabolic index level of the selected subjects was analyzed. The CMI = TG (mmol/L)/HDL-C(mmol/L) × WHtR, triglyceride (TG), high density lipoprotein cholesterol (HDL-C), and waist to height ratio (WHtR) were measured.

The article "Significance of Cardiometabolic Index in Predicting Acute Exacerbation of Stable Chronic Obstructive Pulmonary Disease for Clinical Nursing" was retracted in 2023. Reasons: suspected computer-generated content; unreliable results or conclusions; concerns about the data; concerns about the results or conclusions.

The basic treatment and nursing methods of all patients were basically the same:(1) routine use of ipratropium bromide aerosol and salmeterol ticasone inhalation; (2) TCM comprehensive syndrome differentiation rehabilitation treatment was given. Due to the different constitutions of patients, drug prescriptions were not restricted. In case of an acute exacerbation, TCM intervention should be suspended, and symptomatic and supportive treatment such as anti-infection, bronchodilators, and hormones should be given, and the original treatment should be continued after the condition is stable. Nursing measures are consistent according to the patient's level of education, cognitive understanding ability, and oral expression with a health knowledge manual to patients and their families to introduce the cause of COPD, clinical manifestations, treatment and intervention, clinical outcomes, and other knowledge to help them correctly understand the disease. Use on-site demonstration, pictures, text, and video forms to guide patients to master lip breathing, abdominal breathing, pressure exercise, etc., and give medication guidance. Smoking patients are asked to quit smoking. Criteria for judging acute exacerbation: the clinical symptoms have changed compared with the previous ones, such as cough exacerbation, sputum increase or sputum property change, and dyspnea exacerbation. The range of change exceeds the daily normal variation rate, and due to the change of such symptoms, it is necessary to adjust, increase the use of drugs or further hospitalization.

### 2.3. Statistical Methods

The SPSS20.0 statistical software was used for data processing. Measurement data conforming to the normal distribution are expressed as (*x* ± *s*), while non-normal continuous variables are expressed as median and interquartile spacing (IQR). Categorical variables are represented by constituent ratios. The Spearman correlation test was used to analyze the correlation between variables. Risk factors for acute exacerbation of COPD were analyzed using binary logistic regression. The receiver operating characteristic curve (ROC curve) was plotted to analyze the optimal cut-off value for CMI level prediction of AECOPD, as well as the corresponding sensitivity and specificity. *P* < 0.05 was considered as statistically significant difference.

The article "Significance of Cardiometabolic Index in Predicting Acute Exacerbation of Stable Chronic Obstructive Pulmonary Disease for Clinical Nursing" was retracted in 2023. Reasons: suspected computer-generated content; unreliable results or conclusions; concerns about the data; concerns about the results or conclusions.

## 3. Results

### 3.1. Comparison of Patient General Data

We reviewed data from 63 patients with stable COPD who were admitted to our hospital between January 2021 and December 2021. Demographic, clinical, pulmonary function, and other indicators of the patients are summarized in Table 1. The median incidence of acute episodes in the COPD patients included in the past year was 1. Forty-four patients had ≥1 episode. The cardiometabolic index was 2.33 ± 0.63.

### 3.2. Correlation between CMI and Clinical Data

We analyzed the correlation between CMI and clinical data related to COPD prognosis. The results showed that CMI was positively correlated with the frequency of acute attacks and mMRC score in the previous year (*r* = 0.834. *P* < 0.001), but was negatively correlated with FEV1% PRED (*r* = −0.625; *P* < 0.001) (Table 2).

### 3.3. Risk Factors for Acute Exacerbation of COPD

These data were analyzed using binary logistic regression analysis to determine risk factors for acute exacerbation of COPD. Results showed that CMI measurements were significantly associated with the risk of one or more exacerbations within 1 year (OR 1.596, 95%ci 1.063–2.392), suggesting that CMI is an independent factor of COPD exacerbations (Table 3).

### 3.4. ROC Curve Analysis of CMI Predicting Frequency of Acute Exacerbations

The area under the curve (AUC) of CMI in predicting COPD acute exacerbation was 0.908 (*P* < 0.001) (Figure 1). The cut-off for CMI was 2.05, with 0.864% sensitivity and 0.842% specificity.

## 4. Discussion

In recent years, the status of disease assessment in COPD patient management is becoming more and more important. At present, pulmonary function grading, COPD assessment test score, dyspnea index score, and history of acute exacerbation are mainly used for comprehensive evaluation [7, 8]. However, the above evaluation indexes are highly subjective and require high cooperation degrees of patients, while biological markers are not subject to subjective influence and detection is convenient. It is very significant to find biomarkers that can quantify the severity of disease and predict the prognosis of disease. Therefore, it is of great significance to introduce objective biomarkers to evaluate COPD. In this study, CMI was found to be of great significance in predicting acute exacerbation in stable COPD patients.

COPD is caused by various pathogenic factors that stimulate airway and lung tissue, causing epithelial cell damage, releasing a large number of reactive oxygen species (ROS) and active nitrogen species (RNS), inhibiting the intracellular glutathione (GSH) system. Oxidative/antioxidant balance is broken, resulting in systemic oxidative stress, characterized by increased serum inflammatory markers, including CRP, IL-6, and TNF-*α* [9–12]. Previous studies on biomarkers of acute exacerbation of chronic obstructive pulmonary disease mostly focused on inflammatory factors, such as TNF-*α* and IL-6, and rarely involved other biomarkers. A study of 96,378 patients showed that the CMI level was negatively correlated with cardiac function and positively correlated with the risk of cardiovascular disease [13]. In the study of 11,345 participants, CMI level was shown to be an independent influencing factor for future heart disease [14]. Wang et al. also showed that CMI levels were negatively correlated with cardiac function [15]. COPD is a systemic inflammatory disease, whose systemic oxidative stress can lead to a variety of complications. Cardiovascular disease is the most common and important complication, which seriously affects the prognosis of patients. Therefore, about 1/3 of COPD patients die of cardiovascular disease due to the coexistence of the above two factors [16, 17]. This study analyzed the correlation between CMI and clinical data of COPD patients, and found that CMI was positively correlated with COPD acute exacerbation frequency and mMRC score in the previous 1 year, and negatively correlated with FEV1% PRED. These findings suggest that elevated CMI is associated with a poor prognosis in COPD. Binary regression analysis showed that CMI was a risk factor for COPD progression. The underlying molecular mechanism of the prognostic relationship between CMI and CHF remains unclear. Some scholars speculated that CMI was related to the generation of oxygen free radicals and the oxidation of lipids and nucleic acids [18, 19].

The article "Significance of Cardiometabolic Index in Predicting Acute Exacerbation of Stable Chronic Obstructive Pulmonary Disease for Clinical Nursing" was retracted in 2023. Reasons: suspected computer-generated content; unreliable results or conclusions; concerns about the data; concerns about the results or conclusions.

COPD is a complicated disease with many complications. An acute exacerbation of COPD not only seriously damages lung function and increases the risk of death, but also occupies a large number of medical resources. The United States has taken it as one of the evaluation indicators of hospital medical quality. Early identification of people at high risk of acute exacerbation and appropriate measures can avoid readmission of some patients. In our study, the association between CMI and COPD was reconfirmed, suggesting that a 'patient's CMI level can be used to predict the occurrence of future acute exacerbations. The results suggest that we should not only evaluate 'patients' respiratory function, disease characteristics, and whether there are other complications in nursing evaluation of patients. Nurses also need to evaluate the CMI level of patients. If CMI is higher than 2.05, it indicates that patients have a higher risk of acute exacerbation in the future. Therefore, nursing methods for this group should be different from other patients' and targeted nursing measures should be formulated.

The results of this study not only reinforce previous evidence on the relationship between CMI and COPD outcome but also suggest that CMI is a predictor of COPD acute exacerbation, providing guidance for the development of nursing interventions. Our study also has some limitations. The samples come from a single center and the sample size is small, which may affect the stability of the results.

## Figures and Tables

**Figure 1:** ROC analysis of CMI in predicting the frequency of acute exacerbation of COPD ≥1.

**Table 1:** Characteristics of COPD patients (*n* = 63).

Variables	Mean/N/Median	SD/%/IQR
Demographic		
Age (years-old; median, IQR)	74.00	9.00
Gender (N, %)		
Male (N, %)	37	58.70
Female (N, %)	26	41.30
Smoking status (N, %)		
Smoker	35	55,60
Ex-smoker or nonsmokers	28	44.40
BMI (kg/m2; median, IQR)	22.52	2.09
Clinical		
Course of disease (years; median, IQR)	7.00	3.00
Frequency of acute exacerbation in the past 1 year (median, IQR)	1.00	2.00
Exacerbation frequency≥1	44	69.84
mMRC score (median, IQR)	1.00	1.00
Lung function		
FEV1% pred (median, IQR)	52.76	9.22
CMI	2.33	0.63

**Table 2:** Correlation between GGT and clinical data.

Variables	CMI	
	r	*p*
Frequency of acute exacerbation in the past 1 year	0.834	≤0.001
mMRC score	0.858	≤0.001
FEV 1%pred	−0.625	≤0.001

**Table 3:** Risk factors for acute exacerbation of COPD.

Variables	OR	95% CI	*p*
CMI	1.596	1.063–2.392	0.024

## Data Availability

The data used to support the findings of this study are available from the corresponding author upon request.
